This article has been retracted.

# Genetic Algorithm in Data Mining of Colorectal Images

**DOI:** 10.1155/2021/3854518

**Published:** 2021-10-15

**Authors:** Shou-Ming Chen, Jun-Hui Zhang

**Affiliations:** ^1^Department of Radiology, The Affiliated Hospital of Panzhihua University, Panzhihua, Sichuan 617000, China; ^2^Department of Medical Imaging, Baoji People's Hospital, Baoji, Shaanxi 721000, China

## Abstract

There is currently no effective analytical method in colorectal image analysis, which leads to certain errors in colorectal image analysis. In order to improve the accuracy of colorectal imaging detection, this study used a genetic algorithm as the data mining algorithm and combined it with image processing technology to perform image analysis. At the same time, combined with the actual requirements of image detection, the gray theory model is used as the basic theory of image processing, and the image detection prediction model is constructed to predict the data. In addition, in order to study the effectiveness of the algorithm, the experiment is carried out to analyze the validity of the data of the study, and the predicted value is compared with the actual value. The research shows that the proposed algorithm has certain accuracy and can provide theoretical reference for subsequent related research.

## 1. Introduction

Colorectal cancer is one of the most common malignant tumors in the digestive tract. The 2012 Global Cancer Report of the WHO/IARC (World Health Organization International Center for Cancer Research) shows that colorectal cancer is the third most common malignant tumor in the world and ranks fourth in the cause of malignant tumor death and accounts for about 10% of all cancers. In the same year, there will be an estimated 1.36 million new cases of colorectal cancer, and about 694,000 patients died of the disease [1]. Although the incidence of colorectal cancer is declining in some developed countries [1], the *World Cancer Report* [2] and China's epidemiological studies [3] show that with the aging of China's population, environmental pollution, and changes in living habits, the incidence of colorectal cancer in China is on the rise and there is a trend of rejuvenation. Based on this need, effective monitoring methods are used to improve the effect of colorectal imaging analysis.

Rectal cancer patients account for about 60% of all colorectal cancers in China. With the continuous improvement of surgical methods, the emergence of new treatment methods, and the constant regulation of clinical treatment programs, the recurrence rate of rectal cancer is significantly reduced [4]. However, due to the large base of rectal cancer patients, it is still necessary to further reduce the patient's recurrence rate, improve the prognosis, and improve the survival rate. Accurate preoperative staging of rectal cancer is the main basis for guiding the clinical selection of the best treatment plan (including whether preoperative radiotherapy and chemotherapy, the way of surgery, and the degree of radical cure) and evaluating the prognosis [5]. Inaccurate preoperative staging, whether it is insufficient staging or excessive staging, will have a significant impact on the prognosis of patients.

The American Cancer Association (AJCC) revised the latest TNM staging for rectal cancer in 2010 [6] (determining the T stage according to the depth of intestinal wall infiltration of the primary tumor, the number and distribution of lymph node metastasis to determine the N stage, and whether there is a distant metastasis to determine the M stage), which provides a reliable theoretical basis for preoperative staging of rectal cancer. However, accurate preoperative staging of rectal cancer is still a hot and difficult point in clinical and imaging studies. At present, preoperative T and M staging of rectal cancer can be accurately judged by CT, intrarectal ultrasound, MRI, PET, etc. However, there are many reasons for causing lymphadenopathy around the rectum. Therefore, routine examination based on morphological changes is difficult to make accurate judgments on whether it is benign and malignant, and the accurate evaluation of regional lymph node properties is the biggest challenge for preoperative staging of rectal cancer [7]. Therefore, it is of great significance to study and explore the methods and techniques for accurately determining the nature of rectal cancer regional lymph nodes before surgery to guide the clinical diagnosis and treatment of rectal cancer. There are limited methods of preoperative examination for rectal cancer. Rectal examination is simple and easy and is the most important method for the diagnosis of rectal cancer. It is also the primary examination and diagnosis step for rectal cancer. Therefore, 40%-80% of rectal cancer can be touched during digital rectal examination [8].

Digital rectal examination can provide a preliminary understanding of rectal cancer and its surroundings. However, most of the lymph node metastases of rectal cancer have been in the advanced stage of the disease, and it is impossible to examine rectal cancer with a higher position. Therefore, the clinical examination has limited value in evaluating the regional lymph nodes of rectal cancer. The results of the study of Hardy et al. [9] show that the accuracy of lymph node metastasis by experienced doctors is only 67%. At the same time, the use of digital rectal examination results is not reliable, and it has a great correlation with the experience of the examiner, so it is not used to evaluate regional lymph nodes of rectal cancer. Colonoscopy has been widely used in clinical practice and is the most effective method for the diagnosis of rectal cancer. Moreover, it can directly observe the situation in the intestinal lumen. At the same time, tumor tissue can be taken for pathological examination and partial lesion removal (small lesions, polyps, etc.), which plays an important role in the early diagnosis, treatment, and prevention of rectal cancer. However, colonoscopy not only has many contraindications but also has many shortcomings, such as the risk of perforation and bleeding, the inaccurate positioning of the tumor, and the inability to observe the extraluminal infiltration and regional lymph node metastasis of the tumor, so it cannot be used for the evaluation of regional lymph node staging of rectal cancer.

At present, imaging examination is the main method for evaluating rectal cancer before surgery. The traditional X-ray examination (barium enema, gastroenterology enema contrast) is to display the contour of the digestive tract by introducing the contrast agent into the digestive tract, indirectly observe the anatomy and function of the digestive tract, which can identify the location, gross pathological type, and extent of the tumor, and understand and eliminate multiple primary lesions of colorectal cancer. Moreover, its price is low, and the operation is simple and easy, so it has great clinical value for the diagnosis of rectal cancer. However, it cannot make an objective evaluation of the size of rectal cancer, the degree of extraluminal infiltration, and the surrounding tissue structure. Therefore, an X-ray examination is used as a supplement or replacement only in the case of unsatisfactory colonoscopy or colonoscopy and not as a basis for the diagnosis of rectal cancer. When judging the benign and malignant lymph nodes in rectal cancer, other imaging methods are based on morphological changes such as the lymph node size, morphology, margin, and density/signal/echo, such as conventional abdominal pelvic CT, pelvic MRI/intrarectal MRI, and intrarectal ultrasound (ERUS). However, there are many causes of lymph node enlargement around the rectum, and even small lymph nodes may have metastasis [10]. Therefore, morphological changes alone can easily lead to false negatives and false positives, and the accuracy is not high, which has great limitations on guiding the accurate staging of rectal cancer. In addition, the accuracy of the lymph node size of rectal cancer based on the lymph node size reported in the literature is 55%-71% [11]. With the continuous development of medical imaging, new inspection equipment and technology have emerged, and functional imaging technology has attracted widespread attention from clinical and imaging workers. Currently, common functional tests include CT perfusion imaging, MRI perfusion imaging, magnetic resonance diffusion-weighted imaging (DWI), superparamagnetic iron oxide- (USPIO-) enhanced MRI, magnetic resonance spectroscopy (MRS), single photon emission computed tomography (SPECT), positron emission tomography (PET), and PET/CT. These can not only provide morphological information of the lesion but also reveal the functional metabolism of tissues and organs at the cellular and molecular levels [12].

According to the above analysis, at present, there is no effective analysis method in colorectal image analysis, which leads to certain errors in colorectal image analysis, and some interference factors directly affect the diagnosis results. Based on this, based on the genetic algorithm, this study explores the mining methods that can obtain effective information from the influence of colorectal cancer and promote the further improvement of the diagnosis of colorectal cancer.

## 2. Research Method

### 2.1. GM(1, 1) Model

In the early 1980s, Professor Deng Julong proposed the theory of gray systems. The theory is based on a small-sample, poor-information, and uncertainty system that contains both known information and unknown or unascertained information. The algorithm mainly extracts valuable information from the production and development of some known information and realizes the correct description and effective monitoring of the system's operating behavior and evolution law. Moreover, it finds the law of the data from the chaotic, finite, discrete data and then establishes the corresponding gray model for prediction. GM(1, 1) is an important part of the gray system theory, and it is also the most widely used prediction model. Moreover, its core idea is to determine the best fit curve of a point group generated by the accumulation of the original sequence of the system [13].

Assuming that *X*^(0)^ = (*x*^(0)^(1), *x*^(0)^(2), ⋯, *x*^(0)^(*n*)), *X*^(1)^ = (*x*^(1)^(1), *x*^(1)^(2), ⋯, *x*^(1)^(*n*)) exists,

(1) $$\begin{array}{c} X^{\left(0\right)}\left(k\right)+{ax}^{\left(1\right)}\left(k\right)=b, \end{array}$$

is called the original form of the GM(1, 1) model.

In equation (1), *X*^(0)^(*k*) is the determined output and *b* is the equivalent input obtained by calculation.

Assuming that *X*^(0)^ and *X*^(1)^ are as defined above, then *Z*^(1)^ = (*z*^(1)^(2), *x*^(1)^(3), ⋯, *x*^(1)^(*n*)). Among them, *z*^(1)^(*k*) = (1/2)(*x*^(1)^(*k*) + *x*^(1)^(*k* − 1)). We call that

(2) $$\begin{array}{c} x^{\left(0\right)}\left(k\right)+{az}^{\left(1\right)}\left(k\right)=b, \end{array}$$

is the basic form of the GM(1, 1) model.

The meaning of the symbol GM(1, 1) is the gray model of an order (Order) and a variable (Variable). In the GM(1, 1) model, the time response sequence of *x*^(0)^(*k*) + *az*^(1)^(*k*) = *b* is [14]

(3) $$\begin{array}{c} {\overset{\wedge }{x}}^{\left(1\right)}\left(k+1\right)=\left(x^{\left(0\right)}\left(1\right)-\frac{b}{a}\right)e^{-ak}+\frac{b}{a},\;k=1,2,\cdots ,n. \end{array}$$

In the GM(1, 1) model, the restored value of *x*^(0)^(*k*) + *az*^(1)^(*k*) = *b* is

(4) $$\begin{array}{c} {\overset{\wedge }{x}}^{\left(0\right)}\left(k+1\right)={\overset{\wedge }{x}}^{\left(1\right)}\left(k+1\right)-{\overset{\wedge }{x}}^{\left(1\right)}\left(k\right),\;k=1,2,\cdots ,n. \end{array}$$

It can be seen from equation (3) that the essence of the GM(1, 1) model is to adopt an exponential fitting similar to Ne^*ak*^ for the original data except for the first point. The parameter −*a* in the model is the development coefficient, and *b* is the gray action [15].

There are many models based on the gray system theory. So far, the most common application in the gray prediction model is the GM(1, 1) model, which is also an important part of the gray system theory. For decades, many scholars have conducted a special study on the GM(1, 1) model, which enriches the gray system theory while improving the modeling mechanism and improving the prediction accuracy of the model. Although good results have been achieved in the study of gray prediction models, there are still some mechanistic problems in the gray prediction model that have not been fundamentally solved [16].

In equation (3), there is a boundary value *x*^(0)^(1), but in the process of solving the development coefficient −*a* and the gray action amount *b*, it is independent of the value of the boundary value *x*^(0)^(1). Therefore, the value of the boundary value *x*^(0)^(1) should not be less than the index correction effect of the prediction result. The GM(1, 1) model prediction result is a fitting curve that does not pass the (1, *x*^(0)^(1)) point in the sense of least squares. However, the GM(1, 1) model-defined fit curve must pass the (1, *x*^(0)^(1)) point, which is supported by no theoretical basis [17].

The GM(1, 1) model follows the least squares method to estimate the development coefficient −*a* and the gray action *b*. That is, *a* and *b* satisfy

(5) $$\begin{array}{c} \underset{a,b}{\min}\overset{n}{\underset{i=1}{\sum }}{\left[{\overset{\wedge }{x}}^{\left(0\right)}\left(i\right)-x^{\left(0\right)}\left(i\right)\right]}^{2}. \end{array}$$

In the prediction of the amount of image inspection, we pay more attention to the minimum relative error of the prediction results, that is,

(6) $$\begin{array}{c} \underset{a,b}{\min}\left[\frac{1}{n}\overset{n}{\underset{i=1}{\sum }}\frac{\left|{\overset{\wedge }{x}}^{\left(0\right)}\left(i\right)-x^{\left(0\right)}\left(i\right)\right|}{\left|x^{\left(0\right)}\left(i\right)\right|}\%\right]. \end{array}$$

Therefore, *a* and *b* obtained according to the least squares method are not the best results.

### 2.2. Optimization of the Image Inspection Quantity Prediction Model GM(1, 1)

According to the above analysis of the GM(1, 1) model, firstly, we can add a correction value *ε* to the boundary value of the optimized GM(1, 1) model. That is, the time response sequence of *x*^(1)^(1) = *x*^(0)^(1) + *ε* in the GM(1, 1) model is set to [18]

(7) $$\begin{array}{c} {\overset{\wedge }{x}}^{\left(0\right)}\left(k\right)=\left(1-e^{a}\right)\left(x^{\left(0\right)}\left(1\right)+\varepsilon -\frac{b}{a}\right)e^{-a\left(k-1\right)}. \end{array}$$

Secondly, the range of *a*, *b*, and *ε* is estimated according to the GM(1, 1) model, and the objective equation of equation (8) is constructed, and the quantum genetic algorithm (QGA) is used to solve the parameters.

(8) $$\begin{array}{c} f\left(a,b,\varepsilon \right)=\underset{a,b,\varepsilon }{\min}\left[\frac{1}{n}\overset{n}{\underset{i=1}{\sum }}\frac{\left|{\overset{\wedge }{x}}^{\left(0\right)}\left(i\right)-x^{\left(0\right)}\left(i\right)\right|}{\left|x^{\left(0\right)}\left(i\right)\right|}\%\right],\\ a_{\min}\leq a\leq a_{\max},\\ b_{\min}\leq b\leq b_{\max},\\ \varepsilon_{\min}\leq \varepsilon \leq \varepsilon_{\max}. \end{array}$$

Quantum genetic algorithm (QGA) is a product of the combination of quantum computing properties and genetic algorithms and is a probabilistic evolutionary algorithm proposed by K.H. Han in 2000. The quantum genetic algorithm introduces the quantum state vector expression into the genetic coding and uses the quantum logic gate to realize the evolution of the chromosome so that the quantum genetic algorithm has a richer population than the traditional genetic algorithm and achieves better convergence than the traditional genetic algorithm. In addition, quantum genetic algorithms are based on the representation of quantum state vectors. Moreover, it uses qubits to encode chromosomes so that one chromosome can express the superposition of multiple states and use quantum logic gates to realize chromosome variation and intersection, thus achieving the optimal solution of the target [19].

Quantum genetic algorithms use qubits to encode chromosomes, and it encodes the following.

Assuming $\left[\begin{array}{c} \alpha \\ \beta \end{array}\right]$ is a qubit, $\left[\begin{array}{cccc} \alpha_{1} & \alpha_{2} & \cdots & \alpha_{n}\\ \beta_{1} & \beta_{2} & \cdots & \beta_{n} \end{array}\right]$ is a qubit and |*α*_*i*_|^2^ + |*β*_*i*_|^2^ = 1,  *i* = 1, 2, ⋯, *n*. Then, equation (9) is the *j*-th individual *X*_*j*_′ of the *t*-th generation.

(9) $$\begin{array}{c} X_{j}^{\prime }=\left[\begin{array}{cccc} \alpha_{1}^{t} & \alpha_{2}^{t} & \cdots & \alpha_{n}^{t}\\ \beta_{1}^{t} & \beta_{2}^{t} & \cdots & \beta_{n}^{t} \end{array}\right]\;\left(j=1,2,3,\cdots ,N\right). \end{array}$$

The quantum genetic algorithm uses a quantum revolving gate to perform the mutation operation, and its encoding method is as shown in

(10) $$\begin{array}{c} \left[\begin{array}{c} \alpha_{i}^{\prime }\\ \beta_{i}^{\prime } \end{array}\right]=\left[\begin{array}{c} \cos\left(\Delta \theta_{i}\right)-\sin\left(\Delta \theta_{i}\right)\\ \sin\left(\Delta \theta_{i}\right)\cos\left(\Delta \theta_{i}\right) \end{array}\right]\times \left[\begin{array}{c} \alpha_{i}\\ \beta_{i} \end{array}\right]. \end{array}$$

Therefore, the algorithm flow of optimization of the image inspection quantity prediction model GM(1, 1) is as follows (Figures 1):

1. The GM(1, 1) model is built, and the range of *a*, *b*, and *ε* is estimated
2. The objective equation *f*(*a*, *b*, *ε*) is constructed
3. The population *Q*(*t*_0_) is initialized. Moreover, it is assumed that the total population is *n*, and *n* is binary coded to generate chromosomes encoded in qubits
4. A measurement is performed on each individual in the initial population *Q*(*t*_0_) to obtain a corresponding binary solution set *P*(*t*_0_)
5. The fitness of each determined solution is evaluated by the fitness function
6. Optimal individuals and corresponding fitness are recorded
7. It is judged whether the calculation process can be ended, and if the end condition is satisfied, it is exited; otherwise, the calculation is continued
8. Each individual in the population *Q*(*t*) is subjected to a measurement to obtain a corresponding binary solution set
9. The quantum revolving gate *U*(*t*) is used to perform update and mutation operations on individuals to obtain new populations *Q*(*t* + 1)
10. Optimal individuals and corresponding fitness are recorded
11. The number of iterations *t* is incremented by 1, and the algorithm returns to step (5)
12. *a*, *b*, and *ε* are substituted into the time response sequence of the modelGM(1, 1)
13. The restored value is solved

## 3. Results

The participants include 50 patients with colorectal adenocarcinoma who underwent colorectal adenocarcinoma resection and underwent abdominal pelvic perfusion scan before surgery and were confirmed pathologically as a colorectal adenocarcinoma from January 2018 to December 2018.

The standard constraints are as follows. (1) During CT examination and before surgery, the patient did not have any antitumor treatment. (2) The patient had no history of allergy to iodine contrast agents and signed informed consent. (3) The patient has no serious heart, lung, liver, kidney, and other diseases. (4) The patient is in good general condition and can cooperate with the entire examination process. (5) The patient has no contraindications for antispasmodic drugs (such as prostatic hypertrophy and glaucoma). (6) The patient does not currently have hyperthyroidism. (7) The patient had not had gastrointestinal angiography within 1 week before CT examination and did not take metal-containing drugs. (8) The postoperative pathological data of the patient was recorded in complete detail.

All patients required a less slag diet within 2 days prior to the exam, and the patient required fasting the night before the exam. The body mass was measured to determine the amount of contrast injection. 30-90 minutes before the examination, the patient orally administered 1500 ml 2.5% mannitol until the contrast agent reached the rectum, thereby allowing the gastrointestinal tract to fully expand. 15 minutes before the scan, the patient's buttock muscle was injected with 10 mg of anisodamine hydrochloride to remove body surface metal objects. Moreover, patients need to have repeated breath-holding training. For patients who cannot adhere to it, we need to keep the patient breathing calmly. Conventionally, the abdominal band is added to reduce abdominal movements and to ensure that the patient is at rest during the scan. In addition, the examination process is informed to the patient, and the patient is informed that a normal reaction such as pain and transient fever occurs when the contrast agent is injected. At the same time, it is necessary to obtain the cooperation of the patient to avoid the patient's respiratory movement due to sudden discomfort.

According to the CT scan image, the tumor position is determined, and the largest level of the lesion is selected. Moreover, with this layer as the center, 8 layers are selected as the target level, and the suspected enlarged lymph nodes in the fat space around the lesion are included as much as possible. Thereafter, 300 mg of I/100 ml of iohexol was injected through the median vein of the elbow at a rate of 4.0 ml/s. When injecting contrast agents, close patient response is required. Once there is an adverse reaction, we need to stop the injection and scan immediately. After the contrast agent was injected, 20 ml of physiological saline was injected at the same rate. The film scanning method was used for the same layer dynamic enhanced scanning, and the 8 s sweep was delayed, and the continuous acquisition was 40 s, and 320 perfusion images were obtained. Moreover, the *Z*-axis coverage is 4 cm, the layer thickness is 5 mm, the average scanning interval is 1.0 s, and the scanning parameter is 120 kV, 40 mA.

The acquired perfusion data is transferred to the GE Advantage Workstation 4.3 for viewing images. Whether the lesion is located in the observed scan plane is correct, and whether the lesion position is too large is judged to select the eligible case. The body tumor perfusion software in the preinstalled Perfusion 3.0 software package was then applied for data processing. Thereafter, the threshold range is set to -200 to 120 HU to remove images of tissues such as bone, fat, and air. The first target plane without any enhancement is selected as the basal plane, the plane of the most obvious phase is selected for lesion enhancement, and the abdominal aorta, external iliac artery, or femoral artery is selected as the input artery. After that, the Region Of Interest (ROI) is manually depicted. The ROI is selected at the largest level of the tumor and avoids the edge of the tumor, the markedly enhanced blood vessels, and the necrotic cystic changes and calcifications within the mass, avoiding the effects of partial volume effects. After that, the solid part of the tumor is selected, and the area contains the entire tumor as much as possible (Figures 2 and 3). The perfusion software can automatically analyze the time-density curve (TDC) of the target artery and lesion ROI, the CT perfusion pseudocolor map of this level, and a series of perfusion parameter values such as blood flow (BF), blood volume (BV), mean transit time (MTT), and surface permeability (PS).

Image processing is performed on the above image, and on the basis of this, Figures 2 and 3 can be, respectively, shown in the form shown in Figures 4 and 5.

Figure 4 is used for data mining through the algorithm of this study, and the following information is obtained. The patient is male and has rectal cancer. Surgical pathology confirmed that it was a moderately differentiated adenocarcinoma, invading the whole layer; the two margins were not involved in cancer, and no cancer metastasis was found in the lymph nodes of each group, and the rectal wall underwent eccentric thickening.

Figure 5 is used for data mining through the algorithm of this study, and the following information is obtained. The patient is male and has sigmoid colon cancer. Surgical pathology confirmed that it is a highly differentiated adenocarcinoma that invades the muscular layer. Moreover, there was no cancer involvement in the two margins and the anastomosis ring, and no cancer metastasis was found in the lymph nodes of each group, and eccentric thickening occurred locally in the sigmoid colon.

In order to further study the role of the genetic algorithm model in colorectal image data mining, this study takes the role of ADC as an example for analysis.

In this experiment, the number of lymph nodes included in the metastatic group was 19, and the number of metastatic nodules included was 13. Moreover, the maximum short diameter of the metastatic lymph nodes ranged from 6.20 mm to 17.60 mm, 9 cases were round and elliptical, and 10 cases were lobulated and not smooth. The T2WI fat suppression is a high signal, and the short diameter of the metastatic nodules is 2.10 mm~7.80 mm, which is round or oval, and the boundary is smooth. FST2WI fat suppression is a high signal, and malignant lymph nodes and metastatic nodules are high signals on DWI. The measured ADC values of malignant lymph nodes were 0.80 ± 0.18 × 10^−3^ mm^2^/s, and the metastatic nodule ADC values were 0.78 ± 0.25 × 10^−3^ mm^2^/s, and *p* = 0.80 > 0.05, so the difference was not statistically significant. The comparison between the two groups is shown in Table 1.

The collected test image results are shown in Figure 6.

Image processing is performed on the above image, and the result is shown in Figure 7.

## 4. Analysis and Discussion

Local lymph node metastasis (paraspinal lymph nodes, mesangial lymph nodes) is the most common metastatic pathway for colorectal adenocarcinoma. Therefore, CT perfusion examination of colorectal adenocarcinoma can additionally provide hemodynamic status of regional lymph nodes of colorectal adenocarcinoma in the scan range and indirectly evaluate its angiogenesis. However, there are few reports on the evaluation of regional lymph nodes in colorectal adenocarcinoma by CT perfusion imaging. Compared with tumors, the size of lymph nodes is smaller, and it is more susceptible to intestinal peristalsis, respiratory movement, and partial volume effect. Therefore, this study only selected the largest metastatic lymph node in patients with lymph node metastasis as the “target” lymph node. A total of 19 patients with lymph node metastasis were confirmed by postoperative pathology in this group of data. Among them, 1 case of metastatic lymph nodes was not included in the perfusion scan range, 1 case of lesion position shift in the scan plane due to intestinal peristalsis was too large, and 1 patient's perfusion parameters could not be calculated, so the patient was not included in the study. Moreover, the data standard deviation of this group is large. At present, some scholars use CT perfusion imaging technology to evaluate the nature of lymph node lesions in the neck, axilla, inguinal region, mediastinum, etc., but the results are very different. Therefore, CT perfusion can provide information on blood perfusion of lymph nodes, but the value of evaluating lymph node properties remains to be further studied.

In this study, a genetic algorithm is used as the basic algorithm of data mining, and the detection result has certain superiority compared with the traditional detection algorithm. The predictive performance of image inspection is superior for several reasons. First, the GSVR model of image inspection fully utilizes the preprocessing of data in the gray model, reduces the randomness of the data, increases the regularity of the data, and is more consistent with the nonlinear mapping characteristics of the support vector machine. These make the support vector machine converge more quickly. Second, if the parameters are not properly selected, the support vector machine will be overfitting or underfitting. In this study, the detection function can determine the appropriate parameters to predict the amount of image examination. Furthermore, the GSVR model minimizes structural risk without minimizing training errors and better solves problems such as small samples, nonlinearity, overfitting, dimensionality disasters, and local minima. Therefore, its generalization and promotion ability are excellent.

The genetic algorithm has obvious advantages in the diagnosis and prognosis of colorectal cancer compared with the traditional imaging examination. With the development of new technologies, genetic algorithms are playing an increasingly important role, but they also have certain limitations. Different histological subtypes in colorectal cancer patients also have certain differences in radioactive uptake. Moreover, colorectal cancer containing mucus components may be false negative, and the degree of mucus concentration in tumors is related to the mucus content in tumor cells. The lesser the mucus component, the lesser the amount of mucus ingested, and there is even no significant radioactive concentration. In the diagnosis of postoperative recurrence of colorectal cancer patients, the increase of radioactive intake may be caused by postoperative anastomotic stomatitis, intestinal polyps, intestinal physiologic uptake, and other benign lesions, causing false positives. In addition, in terms of lung metastasis, increased radiation intake may be affected by benign lesions such as tuberculosis and inflammation, causing false positives. Firstly, the metastasis of rectal cancer is slightly different from the metastasis of other parts of the colon. The special venous return system in the lower part of the rectum can cause solitary lung metastasis without liver metastasis, which is difficult to distinguish from single lung nodules. With the application of genomics in the prognosis assessment of colorectal cancer patients, how to label more specific probes at the molecular level will be an opportunity and challenge for the development of nuclear medicine. Secondly, in the upsurge of tumor heterogeneity research, the genetic algorithm plays an important role as a good means of tumor heterogeneity research.

## 5. Conclusion

Based on the genetic algorithm, this study explores the mining methods that can obtain effective information from the influence of colorectal cancer and promote the further improvement of the diagnosis of colorectal cancer. The quantum genetic algorithm is based on the representation of quantum state vectors. It uses qubits to encode chromosomes, allows one chromosome to express multiple states, and uses quantum logic gates to achieve chromosome variation and intersection, thus achieving the optimal solution of the target. At the same time, in this study, according to the CT scan image, the tumor position was determined in the image processing, and the largest level of the lesion was selected. Moreover, with this layer as the center, 8 layers are selected as the target level, and the suspected enlarged lymph nodes in the fat space around the lesion are included as much as possible. In addition, this paper designs a control experiment for analysis. The research results show that the genetic algorithm is used as the basic algorithm of data mining. The detection results have certain advantages over the traditional detection algorithms and can be gradually applied to the clinical detection of colorectal effects.

## Figures and Tables

**Figure 1:** GM(1, 1) control chart.

**Figure 2:** Tumor scan mark image.

**Figure 3:** Image of tumor ROI.

**Figure 4:** Image of tumor scan marks after image processing.

**Figure 5:** Image of cancer ROI after image processing.

**Figure 6:** Detection image of colorectal cancer.

**Figure 7:** Detection image of colorectal cancer after image processing. The (a–d) obtained by the algorithm of this study are, respectively, expressed as follows. (a) The sigmoid wall is thickened, about 10-13 mm thick, the intestinal wall is intact, and the T1WI is low. (b) T2WI fat suppression is a high signal. (c) DWI is a high signal, and the intestinal wall is intact. (d) ADC diagram shows a low signal.

**Table 1:** Comparison of ADC values between malignant lymph nodes and metastatic nodules.

Group	Number	ADC values (×10^−3^ mm^2^/s)
Malignant lymph nodes	19	0.80 ± 0.18
Metastatic nodules	13	0.78 ± 0.25
*p* = 0.80		

## Data Availability

The data used to support the findings of this study have not been made available because we did not obtain permission for data sharing from the data provider.
